# Exploring the interconnection between international crude oil and silver rates volatilities: Novel evidence from the COVID-19 pandemic

**DOI:** 10.1016/j.heliyon.2024.e34545

**Published:** 2024-07-14

**Authors:** Lei Zhou, Zhimin Gong, Lihui Tian, Zaibi Chen

**Affiliations:** a School of Economics and Management, Hunan University of Science and Engineering, Yongzhou, 425199, China; b Business School of Xiangtan University, Xiangtan, 411105, China; c College of Economics and Management, Hunan University of Arts and Science, Changde, 415000, China; d Wuzhou University, China

**Keywords:** Silver price volatility, Oil prices volatility, China stock exchange, Econometric model

## Abstract

Several research studies globally focus on the volatility of gold and oil prices, neglecting an examination of silver price volatility in relation to other market commodities. The current Covid-19 pandemic has led to various uncertainties and fluctuations in financial and stock exchange markets, yet existing literature primarily concentrates on individual product rates rather than combined rate changes. Our study aims to bridge this research gap by analyzing the relationship between oil rates, silver rates, oil rate transitions, and silver rate transitions on the security exchange in China from 1990 to 2022, using the ARDL approach and Nonlinear ARDL for a comprehensive assessment. The findings reveal a significant impact of silver and oil rates on China's security exchange in the future, with the negative effects of oil rate changes and a positive effect of silver rate transitions. In the short term, oil and silver rates play a crucial role in influencing China's security exchange, highlighting the importance of monitoring these trends for investors. It is recommended that investors respond prudently to market transitions, particularly by considering silver as a secure option during times of uncertainty, while policymakers should implement appropriate measures to manage the rapid fluctuations from oil to the security market.

## 1 Introduction

Extreme unpredictability reduces funding and increases stockholders' thoughts, causing asset allotment and portfolio down arrangements, a massive provocation for equity investors, portfolio managers, traders, and hedgers. At times of high unpredictability, the integration of security markets and dependence get hype, as the decrease in the golden time of heterogeneity forces the funders to find various speculation chances for administering funds. Silver and oil are valuable products that are unavoidable for the global financial state and have recently been formulated together with the funder's portfolio equity [1]. Oil is a moving commodity. Moreover, the rate transition gives adequate facts for predictable products and rates of economic quantities [2]. Conversely, silver is frequently regarded as an emergency resource [3]. To extend current portfolios of equity, funders continually change from silver to oil or join them [4]. In fact, in the present era, concern about silver, as well as oil, has been described through expanded transition as well as turmoil as a means of the focus of saving ideas considerations (e.g., because of the increase in oil in 1990, 2014 till 2016 summers collision in oil rates and food issues of 2006). Consequently, short logic of the way facts are shown and told among the oil, silver as well as security markets may assist funders in order to take endangered administration and sound decisions for portfolios [5].

The unpredictability of products and economic environments increased in 2019 due to the coronavirus's rapid spread [6]. Administrations have been focused on establishing boundaries (for instance, nation and territory isolations). The number of causalities and confirmed cases has increased, resulting in financial outcomes, preserving migration, compelling social isolation, and stopping business operations. As an extreme case, China's finances decreased by 6.8 % at the start of 2020, the start of GDP quarterly figures. Security markets begin to decline as COVID-19 instances spread rapidly, with equity funders and product investors growing riskier because of the acute rise in studies and causalities [7]. The association between public health and the share exchange conundrum is supported by findings that health news has a favourable influence on the predictability of awaiting stock returns [8]. [9] asserts that the COVID-19 distribution affects the reliance structure of the endangered-return nexus. A study by ----examined that the current global health crisis has made portfolio management more difficult than in the past due to the recent negative effects of recurrent economic issues, federal unrest, and import-export disputes between the US and China. These factors have increased financial instability and spillover effects. The corona-19 spread substantially impacts the economic units and the actual economy, raising uncertainty [10]. In April 2020, crude Oil (US benchmark) (WTI) decreased by $37 per barrel. This resulted from a sharp decrease in global demand when financial activity was notably sluggish due to lockdowns in nearly all major nations.

The whole first half of 2020 is expected to expand by 30 %, according to the US International Renewable Energy Agency. In comparison, fluctuations in petroleum prices are detrimental to world finance. Factory production and silver prices decreased during the outbreak, indicating an increasing positive potential. According to theory, the prices of silver, oil, and stocks all move in unison, with stock performance influenced by commodity news. Changes in crude petroleum rates impact discount rates and corporate cash flows. The rise in manufacturing values, as well as restricted cash flow caused by the price of oil, affects stock values. Supposedly, several variables, such as expected organizational cash flows, forex marketplaces, economic cyclical, and savings factors, could be responsible for any relationship between share prices and crude oil. More people are purchasing silver as a hedge against dropping equity rates, which raises the metal's price [11]. Silver rates fluctuate instead of being essential for money exchange and transactions [12].

The analysis being conducted today is intended to estimate how shifting silver and oil prices may affect the Chinese security market. There are numerous reasons for the value of the Chinese market. According to Ref. [13], the Chinese are now the globe's most prominent supplier as well as the purchaser of resources, leaving behind the United States. The Chinese overtook the United States as the foremost economic power in the world following the eighteenth Peoples Conference, which took place in the 1990's Nov; the Chinese administration extended the money facility accessible to its registered stakeholders globally (QFII) [14]. Global stakeholders have utilized the Shangai and Shenzhen points of reference. The two countries that use the most oil worldwide are America and China, and China is a significant trading partner for the Group of Oil transferring nations [15]. With a place value of $6.19 trillion in 2022, the Shanghai index is the major security exchange on the planet in Asia-Pacific (after Japan's Nikkei stock indices). The index of Shenzhen, comparably, is ranked fourth (preceding China's security transfer place). Considering that these markets are open to buyers from all over the world, the Chinese global markets are also heavily influenced by foreign disasters. The much more heavily traded resource in the world, oil, influences the stock rates and those of other expensive items. Uncertainty is necessary for economic growth. By examining variations in the prices of silver and oil, one can identify fluctuations in stock rates as products and share place spoilers may occur at any moment, particularly at moments of issues [16].

The country is an important player in the global petroleum sector due to its role as a major purchaser and the highest net exporter of petroleum. Its strong economic growth has also led to the expansion of the Chinese stock market, which has gained the attention of many investors from around the world. As a result, the association between the Chinese share Place and resources values has recently received focus [17] are recent studies that address this issue. Analysis of China has stretched over the stochastic perspective in a few investigations, which concentrate on the antisymmetric effects of oil prices on the share market, disregarding the regressive interrelationships among two variables in the long and short term. According to Ref. [18], the Chinese share place protects investors’ portfolios and provides a haven for them during unstable financial times.

Additionally, we have seen a consistent increase in China's demand for silver over the past few years. High property and stock market uncertainty, rising inflation expectations, and rising worldwide market rates are all factors that have contributed to the massive surge in investment. Comparable to any additional income stream, silver is a viable alternative investment and the best hedge against inflation. It is important to note that the benchmark for silver trading worldwide is the COMEX's three-month silver futures pricing. Such rates will have a critical effect on the Chinese equities markets because China has the fastest-growing silver-containing product market in the world, and silver has become a key component of asset allocation. A significant empirical and theoretical evident relationship between the two variables since we anticipate that China's robust marginal demand for silver will be connected to the global point of comparison for silver rates [19,20].

The study's findings regarding the relationship between fluctuations in international crude oil and silver prices have significant implications for investors and portfolio managers. These insights provide vital information on market dynamics and strategies for managing risk. In today's highly interconnected and unpredictable global financial environment, it is essential to comprehend the correlation between significant commodities like oil and silver and their influence on stock markets. This understanding is vital for making well-informed decisions. The study primarily illuminates the complex correlation between oil and silver prices and the volatility of the stock market. The research reveals the impact of oil and silver price fluctuations on stock prices, considering both immediate and long-lasting effects, through the analysis of data collected over multiple years. Having this knowledge enables investors to predict market fluctuations and make necessary adjustments to their portfolios, thereby reducing risks and maximizing profits. Furthermore, the results offer direction on ways for diversifying portfolios. Historically, investors have sought refuge in gold as a secure and stable investment option in periods of economic instability. Nevertheless, this study emphasizes that silver can be a practical substitute, especially when oil markets experience increased instability. Comprehending the favourable impact of changes in the price of silver on stock prices empowers investors to efficiently distribute their resources, achieving a balance between risk and return in various asset categories.

Furthermore, the study emphasizes the significance of closely monitoring worldwide economic indices and commodities prices. In the present globalized era, occurrences in one region of the world can significantly impact financial markets in other parts of the world. The COVID-19 pandemic is a notable instance, as it has caused significant disruptions to supply chains and economic activity, leading to global impacts on commodity prices and financial markets. Through maintaining awareness and being watchful, investors can modify their approaches in reaction to shifting market circumstances, thus reducing losses and taking advantage of developing prospects. Moreover, the research adds to the ongoing discussion over portfolio optimization and risk management. The study provides a detailed analysis of the connection between commodities prices and stock market volatility by utilizing sophisticated econometric models like ARDL and nonlinear ARDL. Investors can utilize this feature to create advanced risk models and customize their investing strategies according to current market situations. Investors can mitigate their vulnerability to oil price volatility by including silver in their investment portfolios or modifying their asset allocation in response to shifting market conditions. Finally, the reason for undertaking this study is based on its significance in relation to practical investment choices and the development of policies. With the rising complexity and interconnection of financial markets, there is a growing demand for strong empirical research to provide guidance to investors and policymakers. This paper addresses a significant vacuum in the existing literature by presenting new information on the relationship between oil and silver prices and stock market volatility. It also establishes a foundation for future research in this field. In conclusion, the knowledge acquired from this research has the capacity to guide investment approaches, improve the performance of portfolios, and contribute to the durability and effectiveness of financial markets in the future.

This examination is a preliminary study in China, which investigates shifting connections between silver rates and oil rates and their transitions with its security market. This study draws two main conclusions from the literature. As far as the authors are aware, no studies have questioned these associations in a collective or a project using China. Furthermore, the effect of silver rates has not gained more focus, especially in the Chinese market. Hence, this research helped researchers who are striving to observe the connection and adds more detail by guessing this association by taking silver rates and their transitions into observation. Second, we used ARDL bound testing to estimate the extended relationships between oil rates, silver rates, transitions in silver rates, resources rates, and hare place [21,22]. This method is superior to Johansen Co integration because of its multiple benefits. The Cointegration analysis can be successfully deployed, unlike some other methods for assessing, which includes consideration, despite the fact that the examined changes are incorporated of rank 0, level 1, or a blend of both.

However, if the changes were consolidated to plan 2, Autoregressive Distributed lag structure bound techniques might not be effective. At times, an order of lag regarding the structure will be checked, and we can use the conventional weighted least constraint testing method to look at the cointegration. The indigenousness problem is avoided because of the ARDL technique's use of lag values of change. The model successfully calculates this cointegration link using small samples, and it does so without encountering issues with low forecasting efficiency [23,24]. The parts in the end study will be divided into preceding parts: An audit of pertinent literary works will be presented in part two. An assumed model is used, as shown in Portion Three. This study is ended in Article 4, and the following section evaluates and discusses the use of policies.

## 2 Literature review

The research's literature review portion offers a thorough synopsis of previous studies examining the correlation between commodity prices, specifically oil and silver, and the stock market's performance, with a specific emphasis on the Chinese setting. The researchers skillfully combine important research findings, pinpointing areas that need more investigation and acknowledging their study's reasons.

An important recurring topic in literature is the influence of commodity prices on the stock market dynamics. Prior research has thoroughly investigated the correlation between oil prices and the stock market's performance, yielding varied results about the direction and strength of this correlation. Several studies propose a positive correlation between oil prices and stock prices, suggesting that increasing oil prices can boost economic activity and result in higher stock market returns [25]. However, others argue for a negative relationship, stating that higher oil prices can raise production costs and lower corporate profits, which can hurt stock prices (Xiao et al., 2019). There is a lack of research on the relationship between silver prices and stock market performance, and there is limited empirical data on how one affects the other [11].

Another important area of study is the significance of commodity prices about economic well-being and market sentiment. Academics have extensively discussed the degree to which fluctuations in the prices of goods, namely oil, indicate wider economic patterns and investors' feelings. Increasing oil prices can indicate a rise in demand and economic growth, resulting in higher stock market values [26]. On the other hand, abrupt increases or decreases in oil prices might indicate economic instability or geopolitical danger, leading investors to adjust their investment portfolios appropriately [27]. Nevertheless, research on the relationship between silver prices and their use as economic indicators is scarce. Therefore, it is necessary to do additional investigation to determine the extent to which silver prices might serve as a leading indication of market sentiment [28].

Moreover, the literature review emphasizes the need for a more detailed comprehension of the transmission mechanisms by which fluctuations in commodity prices impact the stock market's volatility. Previous research has mostly concentrated on linear connections between variables. However, recent progress in econometric modelling has highlighted the significance of nonlinear and asymmetric impacts [29]. The effect of changes in oil prices on the stock market's volatility might fluctuate depending on the direction and size of the change. Positive changes have distinct consequences compared to negative changes [11]. Similarly, fluctuations in the price of silver may have unequal impacts on the stock market returns, which can be attributed to the behaviour of investors and the market dynamics [21].

Although the existing literature offers significant insights, several limitations and gaps still need to be addressed. Several research studies have mostly concentrated on well-established markets such as the United States and Europe, neglecting the distinct features and dynamics of rising markets such China. Furthermore, most research has primarily used conventional linear models, overlooking the possibility of nonlinear and asymmetric connections between variables. Moreover, there needs to be more literature on the relationship between silver prices and their influence on stock markets, a noticeable deficiency in the current research field. In addition, prior research has frequently disregarded the influence of additional macroeconomic factors and market fundamentals on stock market volatility. This highlights the need for a comprehensive approach to empirical study, as emphasized by Ref. [30].

Given the limitations and gaps in the existing literature, the authors were motivated to conduct the present study. The study aims to offer new insights into the relationship between oil and silver prices and stock market volatility by utilizing modern econometric approaches and focusing on the Chinese environment. The study seeks to enhance our understanding of commodity market dynamics and provide insights for investment strategies and policy decisions in the global economy by addressing previous literature's limitations and utilizing the Chinese market's unique characteristics.

The impact of resources like oil and silver on the performance of stocks is keenly discussed in the current research [31,32]. These authors further explain that adding investments to owners' wallets offers benefits for asset allocation [33]. conducted a study on the influence of presidential retail policy preconceptions on actual metal rates. As a result, although it was revealed that a federal govt bid was more probable, rates have significantly dropped. If the current regime attempted to control the prices or preserve a pricing maximum by surrendering its stockpiling, a pure speculation onslaught might inevitably occur [34]. examined the nations in case they determined the effect of changes in resource prices and the spike in commodity prices on stock returns and found that there was minimal to no influence from these factors [20]. extensively investigated the cross-sectional information for twenty-one nations to pinpoint crucial elements influencing the need for metal in both tangible and profile forms. Analysis of the study revealed considerable differences between tangible and profile stress. Tangible and profile requirements also differed between wealthy and developing countries. Similar to this, in their investigation of how buyers' opinions are affected by fluctuations in metal and metal prices [35]. realized that buyers were ignorant of a significant link between all these rates. Parallel to this, --, while reviewing data on the Spanish capital market, vehemently disputed the safe-haven qualities of Treasury bonds and silver [36]. asserted that a company's volume and transaction costs affect the number of assets retained in cash. Like other sorts of assets, Silver Prizes could be impacted by financial restrictions [37].

An objective measure of UK enterprises revealed that organizations still reserve funds for both operational and protective purposes. A corporation cannot decide to sell holdings, issue new shares, or even establish rules governing quarterly dividend levels unless Silver Prizes are in a position for mercantile incentives [38]. A business may keep investments in the form of currency as a contingency plan for predicted scenes [39]. The business has money on hand, and it can use it not only to survive hard days but also to stop prospective income streams [40].

Changes significantly influence the propensity to manage earnings in a nation's macroeconomic indicators. There is more macroeconomic economic turbulence, and executives behave more eccentrically [41]. The fundamental reason for this is that they cannot foresee corporation realities. When the words used to describe the settings have steadied, each decision is made regarding how much liquid cash they will keep on hand to satisfy the demands of the business [42]. observed in a different study that companies typically increase the quantity of cash that they keep as a security concept during uncertain times and found that businesses tend to increase the cash they hold as a safety measure during uncertain times. As said by Ref. [43], it is evident that unforeseen responsibility to make situations and unpredictability affect enterprises since they increase the number of liquid assets. Because of this, the business holds onto liquidity ratios that aren't being utilized, and there are even delays in starting to plan investments over a long visit [26]. reported similar conclusions to Ref. [44] study on Indian firms. In periods of substantial uncertainty, Indian firms boosted their Silver Prize according to gender and survey size divides made [45]. Also, maintaining valuable credits in small businesses was shown to be disrupted by uncertainty.

Discrepancies can be expressed in a variety of ways. In a survey by --, civil unrest is shown as a key element influencing many firms' willingness to store assets in cash. They discovered that executives are prepared for a little excess wealth to prevent political abduction when a new political system is evolving [8]. split ambiguity into resolute turbulence and business volatility. They also observed short-term volatility of 30 days and long-term fluctuation, unpredictability with a one-year lag (termed a short-time fluctuation). Wright's research identified two categories of individuals' money-hoarding inclinations. Since this is happening, managers may need to put off new venture investments until high sustainability is achieved.

[26] analyzed the influence of rate flipping on the oil, silver, and share prices in China and the US, often during COVID-19. Their study found that the main drivers of these marketplaces were their shocks in the share prices, and consecutive findings show that the oil market was the factor contributing to and beneficiary of both elevated/low dictatorships of uncertainty. In contrast, the stock and silver marketplaces were the beneficiaries or content creators of ripple effects in the tyrannies of low and high volatility, respectively [46]. investigated the effects of the US equity market prices. The price level was reverting to its lengthy optimum at a minor daily readjustment speed, according to the original stud-y application of the ARDL founder forecasting model [47]. used the VAR-GARCH structure to analyze when the unpredictability of metal prices influenced Chinese share market levels between 1990 and 2022. Their studies showed that fluctuations greatly influence the outcome of China's stock market in spot prices. The varying correlation between oil prices, the share market list, metal values, and transfer values in Mexican countries was determined --.

In opposition to metal rates, which have had a minimal empirical influence on the share markets and minimal benefit on currency values, the research from ARDL estimation revealed that oil rates imposed a favourable influence over share market rates over studied time while a detrimental effect over currency rates. Analysis using Ou pas Cause and effect estimation of the correlations between silver, petroleum products, and stocks with economic pressure revealed two-way causality between silver and oil at both means and variation. The complex association between silver and oil along the five primary share markets—namely, Germany, France, the US, the UK, and Japan—was analyzed by -- to see how the COVID-19 epidemic influenced it. According to the author's findings, substantial linkages between silver, oil, and share prices were found in the COVID-19 era as opposed to optimum conditions. -- investigated to evaluate the conditional variance between pairs of semi and energy output at different quantiles and frequency ranges.

According to the study, markets for non-energy products and energy products have weakly significant relationships at given intervals and frequencies. A few non-energy product markets also have a weakly meaningful relation with the prices of global energy commodity markets. Using a bivariate BEKK-GARCH model, -- used the Shanghai, Karachi, and Bombay share markets to explore the transitional spillover between oil and security market returns before and after difficulties time. The study demonstrated spillover among share market and Oil in Karachi in two directions, Shangai in one direction, and Bombay in combined (monodirectional or bidirectional) directions. Furthermore, there was no discernible change in the outcomes before and after issues regarding spillover effects [[48], [49], [50], [51]]. assessed the portfolio and hedging implications of oil importing and oil exporting countries and the transitional spillovers among security places as well as the market of oil. The delayed variance of the share market and oil price significantly influenced unpredictability in the respective areas, as shown by the analysis of the Garch for rectified comparison groups (cDCC) and cointegration test correlation (DCC).

There are more positive shocks than adverse shocks in an asymmetry assessment. For attacked hedging, stockholders of petroleum nations must own more oil resources, according to an analysis. Neither market interrelations among oil trying to export nor oil-importing nations were found. The BEKK-GARCH model is used too. In Pakistani businesses [52], looked at the shock propagation and unpredictability ripple effects among firm oil reserves and stocks. A variance in spillover from equities to petroleum, as well as from oil to shares, was discovered through analysis. The results of the stock selection showed that the benefits of gas and oil in building a conventional profile are crucial.

Additionally, -- examined earlier studies on the connection between oil price shock prices and concluded that rising prices caused a rise in bond yields [48]. employed a regression technique to examine the association between fluctuations in the price of oil and changes in Chinese equity markets. Their investigation revealed that the importance was favourable in the short run and slightly more significant in a bear market environment. Furthermore [17], investigated how oil price fluctuations and shocks impacted the Chinese share market and brought back five industries. It was summed up as changes profoundly influenced Chinese stock rates.

-- investigated bidirectional correlation and cointegration tests of oil products, worldwide silver, and the share market of India. The analysis discovered a positive and negative connection between such changes and between the silver and oil transformations and the Indian stock industry's unpredictability [49]. investigated whether silver acted as a buffer and place of refuge during the COVID-19 epidemic by looking at 13 Asian stock markets. They observed that while Thai and Pakistani had poor safe zones, Indonesians, Tibet, Vietnamese, and Singaporeans had robust safe havens provided by silver. However, considerable research has looked at how shifts impact stock market performance in the price of oil and oil rate migrations across various countries or groupings of countries. According to Ref. [53] and other scholars, though, the effect of silver prices or the silver rates unpredictability indexes on the stock markets has gotten very little attention. We were unable to find a study that looked into the effect of silver and fuel prices, as well as the inferred shifts among them, in the sense of any particular country, to the greatest of our knowledge, and although research on the relationship between inferred silver rate transitions and implied oil rate transformation with equity markets have been performed.

Due to the apparent immense effect that cost instability has on investments in stocks and the prices at which these products are transacted worldwide, it is beneficial that this research discusses how petroleum or metal pricing and fluctuations in those prices affect the Chinese financial markets. Rising volatility in the price of oil and silver serves as a warning and keeps producers and shareholders aware of the potential hazard. As a result, knowing how the rate transitions for these two products operate helps us better understand the stock and finance sector and our economic standing. Furthermore, prior research tended to ignore the awareness of the unforeseen link between such alterations over the long term in favour of calculating the consequences of these changes on share price activity [54]. Thus, as stated in the introduction section, our research makes an essential contribution to the literary works because it uses the ARDL bound test strategy, along with NARDL and asymmetric causality analysis, to approximate the lively affiliation among silver and oil rates also shifts in the goods’ rates Chinese share market. This approach has several benefits instead to traditional causality and Assumptions.

## 3 Data and research method

### 3.1 Data and model specification

The empirical model in this scenario considers stock market values as the regression coefficient and fluctuations in oil, gold, and share market rates to be the explanatory modifying factors. Our study design is specifically defined by its mathematical formalism in Eq (1):

(1) SP=(oilrates,Silverrates,OilVolatility,SilverVolatility

The form of the econometric structure can be chalked out as Eq (2):

(2) $$sp_{t}=\alpha_{0}+\beta_{1}oil_{t}+\beta_{2}silver+\beta_{3}oilvolt_{t}+\beta_{4}silvervolt_{t}+\varepsilon_{t}$$

Where: t = time; Sp = Share Options Indicator; Oil = Oil Ratings; silver = Silver Ratings; silvervolt = Silver Rates Variability Index; oilvolt = Oil Rates Variability Index. It shows the Chinese share market; we selected the CSI300 index. The three hundred most beneficial and actively purchasing equities on Shanghai and Shenzhen share trade make up this capitalization-weighted index. This index represents approximately 60 percent of the total enterprise value. The Federal Reserve provided financial data that we used to assess the data, and we used crude oil rates to calculate oil prices (dollars per barrel). The pricing data, which is displayed as USD per unit weight, was provided by the World Silver Council. The unpredictability of gold rates is assessed using the GVZ indicator, and the instability of petroleum rates is evaluated using the OVX indicator and the average price range. GVZ and OVX are recognized as indexes since they reflect information asymmetries based on past volatility data and shareholder predictions for upcoming market issues [55]. These two lists' data, which span the months of September 1990 and Dec 2022, were obtained from the CBOE's official site [33]. The logarithmic form expresses the changes to enhance the financial statement.

### 3.2 Autoregressive distributed lag structure bound Co integration test

The purpose of the study is to learn more about the connection between worldwide metal costs and petroleum values, as well as the interaction between silver value and oil rate volatility with the share market of China. The study calculates a significant connection between the value of silver, its turbulence, the price of oil, its vix, and equities using the ARDL bound method [51]. The founder lays out the lengthy structural activity of three or more socioeconomic changes. Using long-term error, the co-integrating formula is considered in the error correction model once nonlinearity among variables has been identified (also called correction of errors). It indicates how swiftly things alter over time, demonstrating the institution's stability—using the ARDL strategy has many benefits. The ARDL methodology may be used to answer any enigma, unlike earlier methods of analyzing combination with the machine, irrespective of whether the assessed alterations have a zero cointegration, one order of integration, or a mixture of both. However, if order two was added to the sequence, the ARDL method may not be applied.

Moreover, using a conventional linear regression bounds testing procedure, cointegration is examined after identifying the number of lags of the model (OLS). Thirdly, the ARDL method with lag change helps solve the indigeneity problem. Lastly, if we simulate the co-integrating association with little chunks, the strategy will work better, and worries about poor power will be dispelled [50].

Robert Person was initially used in our inquiry stages, and the first difference is in the KPSS and ADF root unit tests. These techniques ensure that the data is stationary and does not have a third order of integration. The ARDL model is developed in the second stage using the specifications and the AIC (Akaike information criterion). Based on descriptions and AIC, the ARDL model is generated in a second phase (Akaike information criterion). Then, using bounds testing, it is determined whether the reliant and explanatory changes have a founder connection. We computed the UECM (unrestrained error correction mechanism) regressions in the following ways because relevant research is scarce, and there is debate over the direction of the long-term association in Eqs (3), (4), (5), (6), (7):

(3) $$\Delta oil_{t}=\alpha_{0}+\alpha_{1}oil_{t-1}+\alpha_{2}{silver}_{t-1}+\alpha_{3}oilvolt_{t-1}+\alpha_{4}silvervolt_{t-1}+\alpha_{5}sp_{t-1}+\sum_{i=1}^{n}\alpha_{5}\Delta oil_{t-i}+\sum_{i=1}^{n}\alpha_{6}{silver}_{t-1}+\sum_{i=1}^{n}\alpha_{7}oilvolt_{t-i}+\sum_{i=1}^{n}\alpha_{8}silvervolt_{t-i}\sum_{i=1}^{n}\alpha_{9}sp_{t-i}+\varepsilon_{1t}$$

(4) $$\Delta gold_{t}=\partial_{0}+\partial_{1}{silver}_{t-1}+\partial_{2}oil_{t-1}+\partial_{3}oilvolt_{t-1}+\partial_{4}silvervolt_{t-1}+\partial_{5}sp_{t-1}+\sum_{i=1}^{n}\partial_{5}\Delta {silver}_{t-1}+\sum_{i=1}^{n}\partial_{6}oil_{t-i}+\sum_{i=1}^{n}\partial_{7}oilvolt_{t-i}+\sum_{i=1}^{n}\partial_{8}silvervolt_{t-i}+\sum_{i=1}^{n}\partial_{9}sp_{t-i}+\varepsilon_{2t}$$

(5) $$\Delta oilvolt_{t}=\gamma_{0}+\gamma_{1}oilvolt_{t-1}+\gamma_{2}oil_{t-1}+\gamma_{3}{silver}_{t-1}+\gamma_{4}silvervolt_{t-1}+\gamma_{5}sp_{t-1}+\sum_{i=1}^{n}\gamma_{5}\Delta oilvolt_{t-i}+\sum_{i=1}^{n}\gamma_{6}oil_{t-i}+\sum_{i=1}^{n}\gamma_{7}{silver}_{t-1}+\sum_{i=1}^{n}\gamma_{8}silvervolt_{t-i}+\sum_{i=1}^{n}\gamma_{9}sp_{t-i}+\varepsilon_{3t}$$

(6) $$\Delta silvervolt_{t}=\mu_{0}+\mu_{1}silvervolt_{t-1}+\mu_{2}oil_{t-1}+\mu_{3}{silver}_{t-1}+\mu_{4}oilvolt_{t-1}+\mu_{5}sp_{t-1}+\sum_{i=1}^{n}\mu_{5}\Delta silvervolt_{t-i}+\sum_{i=1}^{n}\mu_{6}oil_{t-i}+\sum_{i=1}^{n}\mu_{7}{silver}_{t-1}+\sum_{i=1}^{n}\mu_{8}silvervolt_{t-i}+\sum_{i=1}^{n}\mu_{9}sp_{t-i}+\varepsilon_{4t}$$

(7) $$\Delta sp_{t}=\delta_{0}+\delta_{1}sp_{t-1}+\delta_{2}{silver}_{t-1}+\delta_{3}oilvolt_{t-1}+\delta_{4}silvervolt_{t-1}+\delta_{5}oil_{t-1}+\sum_{i=1}^{n}\delta_{5}\Delta sp_{t-i}+\sum_{i=1}^{n}\delta_{6}{silver}_{t-1}+\sum_{i=1}^{n}\delta_{7}oilvolt_{t-i}+\sum_{i=1}^{n}\delta_{8}silvervolt_{t-i}\sum_{i=1}^{n}\delta_{9}oil_{t-i}+\varepsilon_{5t}$$

Where oil denotes global oil prices, silver denotes silver rates, silvervolt denotes variability in silver values, oilvolt shows variability in the price of oil, and sp denotes the Shanghai share exchange. All of the equations above have the following H0:

$${Oil\;equation\;\alpha }_{1}=a_{2}=a_{3}=a_{4}=0$$

$${Silver\;equation\;\beta }_{1}=\beta_{2}=\beta_{3}=\beta_{4}=0$$

$${OilVolt\;equation\;\gamma }_{1}=\gamma_{2}=\gamma_{3}=\gamma_{4}=0$$

$${SilverVolt\;equation\;\alpha }_{1}=\mu_{2}=\mu_{3}=\mu_{4}=0$$

$${SP\;equation\;\delta }_{1}=\delta_{2}=\delta_{3}=\delta_{4}=0$$

The H0 in the four formulations above accounts for the series' lack of a long-term relationship. The Wald F-test is used to investigate this claim. The Statistical technique and the lower and upper Pivotal values are calculated using the magnitude of the delayed components changes equation. Cointegration expands specified boundary essential ingredient, and statistics F supports it, and vice versa. If the statistic F falls among relevant lower and upper bounds, no conclusions can be made about the outcome. The error term, sometimes called an erroneous redress term, is used to construct the co - integrating equation once the collinearity between modifications has been established. The association's degree of steadfastness is demonstrated in Eq (8).

(8) $$\Delta oil_{t}=\alpha_{0}+\sum_{i=1}^{n}\alpha_{5}\Delta oil_{t-i}+\sum_{i=1}^{n}\alpha_{6}\Delta silvervolt_{t-1}+\sum_{i=1}^{n}\alpha_{7}\Delta oilvolt_{t-i}+\sum_{i=1}^{n}\alpha_{8}\Delta silvervol{t_{t}}_{-i}\sum_{i=1}^{n}\alpha_{9}\Delta sp_{t-i}+\theta ECT_{t-i}+\varepsilon_{it}$$

Where the ECTt-1 sentence denotes how fast stability returns after a little-term shock. We utilized linearity analysis as CUSUMSQ and CUSUM after the assumed analysis, economically reported inside useful bound of five percent displaying firmness and regression resilience formula, and used the quadratic Autoregressive distributed lag model and unequal pattern recognition during the assumed procedure.

### 3.3 ARDL non-linear estimation

The NARDL model may be perceived as less appealing due to its complexity in handling serial correlation, as indicated by the decreased score. In comparison, NARDL outperforms the Criterion structure technique by considering both short- and long-term asymmetries, while the co-integrating structure only focuses on long-term disparities. NARDL's ability to account for both short and long-term aspects enables it to outperform the co-integrating model. Moreover, it distinguishes between the short and long-term effects of changes in predictor variables. These criteria can be evaluated using a regressive barrier VECM or autoregressive vector strategy, but these methods may face challenges due to numerous parameters. The NARDL paradigm does not encounter such issues.

Additionally, the Partial adjustment model, in contrast to other ECM systems, does not require the same level of stationarity across all periods, allowing for flexibility in integrating time series analysis with different orders of integration. Economic data series need to be adaptable. By decomposing independent variables into partial sums of positive and negative values, the NARDL strategy incorporates both long and short anomalies. The approach of breaking down asymmetries considers fluctuations in population size using the partial sum technique. The Hatemi-J (2012) correlation test is employed to evaluate the direction of asymmetry causation, which is crucial for distinguishing the causal relationships of shocks. A normality test (dmax) is typically conducted as the first step to assess the degree of integration of shifting variables. This is followed by determining the optimal lag period for the vector autoregression model based on the available data. The order of the time series regression is then calculated, and the Wald test is applied to identify significant relationships among variables.

## 4 Data analysis and results

Assessments are initially conducted for regression analysis to evaluate the process of sequence integration before proceeding with ARDL testing. It is crucial to ensure accurate results by integrating the series using the ARDL technique, as indicated in Table 2. The identification of unit roots is carried out individually through PP, KPSS, and ADF tests, all conducted at the same level with considerations for step changes, continuity, and constant initial differences. Findings from these tests are presented in Table 1 below. Unlike the KPSS test, both the PP and ADF tests operate under the assumption that the sequence is entirely non-stationary. Results indicate that neither series exhibits second-order integration. In the Var model, the lagged organization of observed events remains apparent, as illustrated in chart two using the AIC criterion, Schwartz threshold, and Hannan-Quinn Akaike Information (HQ) with a maximum lag length of 4. The examination for cointegration assesses whether changes in motions are consistently linked, as shown in Table 3. The founder establishes long-term fundamental co-movements between two or more macro financial changes. Collinearity is crucial in eliminating misleading correlations. When market values are utilized as variables, correlations are observed among multiple stock rates. In essence, any reform initiatives are likely to impact the stock market first, followed by fluctuations in bullion values and oil rates. The significance of the founder is evident at a 10 % statistical level, with silver rate changes being explained by F-values of inventory rates and silver rate volatility ranging between 5 % and 10 %. Long-term parameter predictions from the ARDL bounds test methodology are detailed in Table 4, following unit cointegration and root calculations. Significant influences on the Chinese stock market are observed from all adjustments, whether positive or negative. Silver rates have a negative impact on subsequent factors. Table 4 presents the Estimated Coefficients of the ARDL Long-Term Model.

**Table 1:** An analysis of the root unit.

Unit-root (level)	(ADF)	(PP)	(KPSS)
Oil	−2.132	−2.334	0.795^a^
	0.421	0.410	
Silver	−1.561	−1.564	0.348^a^
	0.673	0.67	
Oilvolt	−4.0571		
	0.336		
Silvervolt	−1.245	−1.675	
	0.679	0.671	
Sp	−0.048	0.094	0.254^a^
Unit-root (1st difference) D(Oil)	−57.567	−57.60	0.067
	0.000^a^	0.000^a^	
D(Silver)	53.81	53.81	0.012
	0.000a	0.000^a^	
D(oilvolt)	−56.75	−55.01	0.07
	0.000^a^	0.000^a^	
D(Silvervolt)	−49.67	−49.67	0.06
	0.000^a^	0.000^a^	
D(sp)	49.56	−49.94	0.062
	0.000^a^	0.000^a^

**Table 2:** Optimum lag results order of selection.

Lag:	LogL:	LR:	FPE:	AIC:	SC:	HQ:
0:	49.342	49.965	2.45E-23	−3.06743	−3.0897	−2.4965
1:	129.633	20.324^a^	7.98E-87	−5.03245	−3.0623	−3.9953
2:	140.639	19.8762	3.01E-22	−2.9976	−5.0463	−3.4298
3:	232.581	19.4376	3.02E-76	−6.0654	−2.0543	−4.5043
4:	249.498^a^	30.6982^a^	3.06E-82	−6.6290^a^	−1.3078^a^	−4.0723^a^

**Table 3:** Bounded cointegration test for ADLS

Dependent variable	Cointegration (H0)	F-test structure of optimal lag	F-test	Result
Oil	$\alpha_{1}=a_{2}=a_{3}=a_{4}=0$	(2,1,2,2)	2.308	No cointegration
Silver	$\beta_{1}=\beta_{2}=\beta_{3}=\beta_{4}=0$	(1,4,4,1)	1.293	No cointegration
Oilvolt	$\gamma_{1}=\gamma_{2}=\gamma_{3}=\gamma_{4}=0$	(4,2,1,4)	1.234	No cointegration
Silvervolt	$\alpha_{1}=\mu_{2}=\mu_{3}=\mu_{4}=0$	(4,2,1,1)	3.554	Cointegration**
Sp	$\delta_{1}=\delta_{2}=\delta_{3}=\delta_{4}=0$	(4,1,2,4)	5.545*	Cointegration*

**Table 4:** Estimated coefficients of the ARDL long-term model.

Outcome -variable (Stock-price)	Coeff:	P-value
Oil	−5.043	0.000
Silver	−3.231	0.008
Oilvolt	−0.098	0.000
Silvervolt	0.071	0.031
Cons	15.689	0.000

Table 1 examines the presence of unit roots in different variables. This analysis utilizes various unit root tests, including Augmented Dickey-Fuller (ADF), Phillips-Perron (PP), and Kwiatkowski-Phillips-Schmidt-Shin (KPSS).

Both oil and silver prices in the level form have unit root features, as shown by their test statistics and p-values across many tests. These variables are likely to be non-stationary and may display trends or gradual changes over time. Similarly, the variables Oilvolt and Silvervolt, which indicate the changes in oil and silver rates, likewise exhibit unit root behaviour in their level form, suggesting that they are not stationary.

However, when examining the initial differences of these variables, a common practice to attain stationarity, all variables exhibit notable negative test statistics and p-values approaching zero in the ADF, PP, and KPSS tests. After using the differencing technique, these variables exhibit stationarity, indicating the absence of unit root properties and making them appropriate for time series analysis.

From an economic perspective, this means that the fluctuations in oil and silver prices, as well as the speed at which these fluctuations occur, are more significant for analysis than the actual levels of these prices. By ensuring stationarity in these initial differences, it becomes possible to examine the correlations between these variables and other economic indicators without the complications caused by non-stationarity problems. Investors and regulators must have a comprehensive grasp of the temporal dynamics of these variables' swings to make informed decisions, particularly in the security exchange realm, since these changes might have substantial consequences. Hence, it is crucial to ensure that the initial differences of these variables exhibit stationarity in order to carry out relevant and dependable econometric research and forecasting within the realm of financial markets.

Table 2 displays the outcomes of selecting the optimal lag order using several criteria. The findings suggest that the optimal lag order differs based on the selection criteria used. By using the AIC criteria, it has been shown that the optimal lag order is 4, which is associated with the lowest value of −6.6290. Similarly, the lag order of 4 produces the lowest values for both the Schwarz Criterion (SC) and Hannan-Quinn Criterion (HQ). When assessing the Likelihood Ratio (LR) statistic, the optimal lag order is determined to be 1, as it corresponds to the maximum value of 20.324. According to the LR criteria, a lag order of 1 is the most suitable for fitting the data. From an economic standpoint, choosing the optimal lag order is of the utmost importance in time series analysis since it dictates the number of previous observations that are taken into account when predicting future values. The variations in lag order selection among criteria emphasize the significance of considering many criteria and selecting the most suitable one depending on the particular context and aims of the research.

When choosing the lag order, there is a balance between the complexity of the model and how well it fits the data. A higher lag order may capture more specific patterns in the data but may also lead to overfitting. On the other hand, a lower lag order may result in underfitting but provides a simpler model. Consequently, researchers and analysts must thoroughly evaluate these factors and choose the appropriate lag sequence that achieves the optimal equilibrium for their investigation.

Table 3 displays the outcomes of the bounded cointegration test for autoregressive distributed lag (ADL) models, investigating the existence of cointegration between the dependent variables and their lagged values. The null hypothesis of no cointegration for oil prices (Oil) is not rejected, suggesting that there is no long-term correlation between oil prices and their previous levels. The F-test value of 2.308 corroborates this.

Similarly, the null hypotheses of no cointegration for silver prices (Silver) and oil rate transitions (Oilvolt) are not rejected. This suggests that there is no long-term link between these variables and their lagged values. The F-test statistics for silver and oilvolt are 1.293 and 1.234, respectively.

However, the null hypothesis of no cointegration for silver rate transitions (Silvervolt) and the security exchange (Sp) is rejected, suggesting that there is a long-term relationship between these variables and their lagged values. The F-test statistics for silvervolt and Sp are 3.554 and 5.545, respectively.

Cointegration, from an economic perspective, indicates a durable state of balance between variables, indicating that they exhibit a synchronized movement over time, even in the presence of short-term perturbations. Within the realm of financial markets, the presence of cointegration between variables, such as changes in the price of silver and the performance of the security exchange, signifies a durable and consistent long-term connection. Investors can utilize this connection to inform their decision-making processes and effectively manage risks.

Nevertheless, the lack of cointegration between variables such as oil prices and their rate transitions indicates that these variables do not exhibit a consistent long-term relationship. This finding could impact investing strategies and portfolio management.

Table 4 illustrates the outcomes of a regression analysis involving the stock price as the dependent variable and independent variables such as Oil, Silver, Oilvolt, Silvervolt, and a constant term (Cons). Each variable is accompanied by its coefficient estimate and corresponding p-value, which signifies the significance of the variable's influence on the stock price. In economic terms, these coefficients indicate the expected variation in the stock price when each independent variable increases by one unit while holding all other factors constant. For instance, the coefficient for Oil is −5.043 with a p-value of 0.000, indicating that a one-unit increase in Oil is associated with a decrease of approximately $5.043 in the stock price, with other variables remaining constant. Similarly, the regression coefficient for Silver is −3.231 with a p-value of 0.008, indicating a negative relationship between Silver and the stock price, although not as strong as that of Oil.

Conversely, Oilvolt has a coefficient of −0.098 with a p-value of 0.000, suggesting a slightly lesser negative impact on the stock price compared to Oil. On the other hand, Silvervolt has a coefficient of 0.071 and a p-value of 0.031, implying a positive relationship with the stock price, albeit weaker than other factors. The constant term (Cons) in the regression equation represents the intercept and forecasts the stock price when all independent variables are zero. In this case, the Cons coefficient is 15.689 with a p-value of 0.000, indicating a substantial and statistically significant effect on the stock price, irrespective of other factors. In conclusion, the regression results offer valuable economic insights into the connections among oil, silver, oilvolt, and stock prices. They aid investors, analysts, and policymakers in understanding the impact of fluctuations in these factors on stock prices and in making informed decisions in financial markets. The corrections made to errors in the ARDL Model (Short-Term) are detailed in Table 5.

**Table 5:** Correcting errors in the ARDL model (short-term).

All changing	d-SP	t-stat
Error correction term	−0.0152***	−1.842
ds(-1)	−1.0507	−1.236
doil(-1)	0.0574***	−1.063
dsilver(-1)	−1.0211	−0.005
dsilver(-2)	0.0134	1.734
dsilver(-3)	0.0530***	3.415
dsilvervolt(-1)	−0.013	−1.543
doilvolt(-1)	0.0032	1.437
Cons	1.000	0.000

Table 5 presents the results of a dynamic regression model that explores the connection between changes in the stock price (SP) and past changes in various independent variables such as d-SP (change in stock price), doil (change in oil price), dsilver (change in silver price), dsilvervolt (change in silvervolt), and doilvolt (change in oilvolt). The model incorporates an error correction term and a constant term (Cons). The statistically significant error correction term (−0.0152) at the 1 % level indicates a long-term equilibrium relationship between the stock price and the independent variables, suggesting that any deviations from this equilibrium are gradually corrected, demonstrating a consistent and enduring link between the variables. While some coefficients for delayed changes in independent variables show statistical significance, others do not. For instance, the statistically significant coefficient for doil(-1) (lagged change in oil price) is 0.0574 at the 1 % level, showing that past changes in oil prices positively affect the current stock price. Moreover, the significance of the coefficients for dsilver(-3) and dsilvervolt(-1) at the 1 % level implies that changes in silver and silvervolt prices from three periods and one period ago, respectively, have a notable impact on the current stock price. Conversely, coefficients like dsilver(-1) and dsilver(-2) lack statistical significance, indicating that fluctuations in silver prices from one and two periods ago do not significantly influence the current stock price. To sum up, these regression results offer valuable insights into the dynamic relationship between stock price fluctuations and changes in other economic variables, aiding investors, analysts, and policymakers in understanding how past fluctuations in oil, silver, and silvervolt prices affect present stock prices, thereby enhancing decision-making in financial markets. A low short-term error coefficient signifies a slow rate of adjustment towards equilibrium. The symbols *, **, and ***, correspondingly represent significance levels of 1 %, 5 %, and 10 %. The Long-term and short-term results of NARDL are presented in Table 6.

**Table 6:** Results of Long-term and Short run of NARDL.

Estimation of Long-term Changing P-value Coefficient		
Oil	−2.995	0.011
dsilvervolt(-1)^+^	1.550	0.124
doilvolt(-1)-	−0.967	0.835
doilvolt(-1)+	−0.889	0.776
Cons	1.000	0.000
Diagnostics Statistics p-value LM test	0.9733	0.608
Silver	−1.223	0.090
Oilvolt	−1.246	0.010
Silvervolt	1.602	0.018
Short Run Estimation dSP(-1)	−0.027	0.000
doil(-1)+	−0.298	0.009
doil(-1)-	−0.089	0.023
dsilver(-1)-	−0.010	0.008
dsilver(-1)+	−1.223	0.006
dsilver(-2)-	−0.099	0.998
dsilver(-2)+	−0.786	0.334
dsilver(-3)-	−0.667	0.076
dsilver(-3) + dsilvervolt(-1)^-^	−1.432	0.088
	0.114	0.678
dsilvervolt(-1)^+^	2.012	0.212
doilvolt(-1)-	−1.025	0.976
doilvolt(-1)+	−0.903	0.813
Cons	1.000	0.000
Diagnostics Statistics p-value LM test	1.065	0.593
Heteroscedastic test	0.8043	0.913
Normality test	0.296	0.513

The table provided above illustrates the impact of independent component lag on the stock market, showing how certain factors can have an immediate influence. For instance, a 1 % increase in the initial difference in oil prices from three days ago is linked to a 5.7 % rise in the SP now, while a 1 % increase in the initial difference in silver rates from the day before results in a 5.3 % increase in the SP today. Other changes listed in the table do not have an immediate effect on Chinese stock rates. Additionally, Fig. 1 showcases CUSUM chart for stable coefficients [Impact of silver volatility (**A**) and impact of oil volatility(**B**)] from 1990 to 2022, while Fig. 2 delves into the long and short-run effects of changes in oil prices [Impact of oil volatility **(A)** and impact of silver volatility **(B)].**

**Fig. 1:** The ARDL model's CUSUM chart for stable coefficients [Impact of silver volatility(**A**) and impact of oil volatility(**B**)] from 1990 to 2022.

**Fig. 2:** The long and short-run effects of changes in oil prices [Impact of oil volatility **(A)** and impact of silver volatility **(B)**].

Table 6 displays the estimated impacts of various independent factors on the dependent variable, likely the stock price, in both the long-term and short-term scenarios. In the long-term analysis, attention is primarily given to the coefficients associated with the independent variables, while the short-term examination focuses on the immediate changes in these variables. Concerning the long-term forecast, The coefficient for Oil is −2.995, with a p-value of 0.011, indicating a statistically significant negative impact on the dependent variable. The variable dsilvervolt(-1) shows a coefficient of 1.550 and a p-value of 0.124, suggesting a positive effect that is not statistically significant. The coefficients for doilvolt(-1)- and doilvolt(-1) + are both negative in value but lack statistical significance. The variable “Cons” serves as the intercept term in the model, with a coefficient of 1.000 and a p-value of 0.000, indicating statistical significance. Diagnostic data, such as the p-value of the LM test, are provided to assess the overall fit quality of the long-term model. For the short-term analysis: The coefficient for the variable dSP(-1) is −0.027, statistically significant at the 1 % level, suggesting a notable impact of past changes in the dependent variable on the current stock price. Fluctuations in oil prices, represented by doil(-1)+ and doil(-1)-, yield varied results. One of the coefficients, doil(-1)+, is statistically significant, while the other is not. Lagged changes in silver prices (dsilver(-1), dsilver(-2), dsilver(-3)) show mixed effects, with some coefficients being statistically significant and others not. Similarly, coefficients for dsilvervolt(-1)+, dsilvervolt(-1)-, doilvolt(-1)+, and doilvolt(-1)- also show a mix of significant and non-significant results. Diagnostic statistics, including p-values for LM tests, heteroscedasticity tests, and normality tests, are provided to assess the overall fit and validity of the short-term model. In conclusion, these estimations offer valuable insights into the connections between independent variables and stock prices, both in the immediate and long term. They serve as crucial tools for investors, analysts, and policymakers to understand the complexities of the stock market and make informed decisions.

### 4.1 Analysis of causality of asymmetric

In the final analysis, chart seven presents a study conducted by Hatemi-J (2012) regarding asymmetric antecedent evaluation. The data in the table illustrates an unconfirmed hypothesis stating that positive changes in silvery, silvervolt, oil, and oilvolt may not necessarily result in favourable changes in SP, and minor changes in silvervolt, oil, and oilvolt do not necessarily lead to negative changes in SP. Following the examination, it can be inferred that a causal asymmetry exists between SP and the other parameter series in the model. This implies that the relationship between SP and the other parameter series is not symmetrical, indicating that the impact of one variable on the other is not reciprocal. However, the influence of SP on the other parameter series may differ from that of the other parameter series on SP. Statistical analysis has brought to light this relationship, which could have significant implications for comprehending the connections between these variables and forecasting their behaviour. Fig. 3 displays The NARDL model's CUSUM chart for stable coefficients [CUSUM of squares (A) and CUSUM (B), while Table 7 showcases the Analysis of Asymmetric causality.

**Fig. 3:** The NARDL model's CUSUM chart for stable coefficients [CUSUM of squares (A) and CUSUM (B)].

**Table 7:** Analysis of Asymmetric causality.

Null hypothesis	Value of test	Crit-value (1 %)	Crit-value (5 %)
Silver^+^ has not caused SP^+^	201.77	18.09	11.50
SP^+^ has not caused Silver^+^	7.65	5.55	3.09
Silver^−^ has not caused SP^−^	126.39	22.77	11.99
SP- has not caused silver-	14.56	13.32	4.09
Oil^+^ has not caused SP^+^	6.76	11.50	4.89
SP^+^ has not caused Oil^+^	203.33	17.09	11.09
Oil^−^ has not caused SP^−^	0.81	21.33	4.76
SP- has not caused oil-	7.33	13.54	4.09
Oilvolt^+^ has not caused SP^+^	12.87	11.40	11.60
SP^+^ has not caused Oilvolt^+^	8.36	15.65	4.99
Oilvolt^−^ has not caused SP^−^	6.77	14.99	3.97
SP- has not caused Oilvolt-	5.89	7.20	4.67
Silvervolt^+^ has not caused SP^+^	8.38	7.67	3.77
SP^+^ has not caused Silvervolt^+^	7.01	6.66	4.95
Silvervolt^−^ has not caused SP^−^	7.34	18.01	4.30
SP- has not caused Silvervolt-	16.36	15.65	4.89

Table 7 displays the findings of the study of asymmetric causality, which investigates the causal connections between various variables at varying degrees of significance. In each case, the null hypothesis is whether there is no causal relationship between the two variables. The test statistics are then compared to critical values at significance levels of 1 % and 5 %.

The test statistic for examining the influence of Silver+ (positive shocks in silver prices) on SP+ (positive shocks in stock prices) is 201.77. This surpasses the crucial value at both the 1 % and 5 % significance levels, demonstrating compelling evidence to reject the null hypothesis. Hence, upward fluctuations in silver prices exert a substantial causal impact on upward fluctuations in stock values.

In contrast, when analyzing the influence of SP + on Silver+, the test statistic is 7.65, which falls below the critical values at both levels of significance. Therefore, based on the available information, we cannot reject the null hypothesis, indicating that positive fluctuations in stock prices do not have a major impact on positive fluctuations in silver prices.

Additional analyses are performed for various combinations of variables, such as Silver− (representing negative shocks in silver prices), SP- (representing negative shocks in stock prices), Oil+ (representing positive shocks in oil prices), Oil− (representing negative shocks in oil prices), Oilvolt+ (representing positive shocks in oil rate transitions), Oilvolt− (representing negative shocks in oil rate transitions), Silvervolt+ (representing positive shocks in silver rate transitions), and Silvervolt− (representing negative shocks in silver rate transitions).

The results offer valuable insights into the direction and significance of causal linkages among various variables, aiding in the comprehension of how shocks in one variable impact another variable in an unequal manner. Comprehending this knowledge is essential for investors and policymakers to efficiently predict and handle the consequences of economic disturbances on financial markets.

## 5 Conclusion and policy recommendations

The impact of the silver and oil sectors on the share market and, subsequently, on the economy is now widely recognized. Various literature emphasizes the crucial role that silver and oil play in establishing a stable foundation and implementing risk management strategies. The connection between the Chinese share market and the silver and oil markets has been acknowledged due to the significant role these commodities hold in the economy. While previous studies focused mainly on historical variability assessments, our study stands out by examining oil and silver prices from September 1990 to December 2022. We explored the relationships between the Chinese share market, silver, and oil, along with their respective variation lists. By developing anticipated variance lists based on choice rates, we were able to reflect investors' expectations for future market dynamics compared to historical rates. These variance measurements, acting as an effective early warning system, offer insights into potential market concerns. Our research, utilizing Ardl Bound testing, quadratic ARDL, and asymmetry causality analytical techniques, indicates that the increasing global prices of silver and oil could have a lasting impact on the share market. This underscores how stock markets tend to decrease as silver and oil prices rise worldwide. Notably, our study found that while fluctuations in oil prices have a long-term negative effect on the Chinese stock market, significant variances in silver prices have a long-term positive impact. These findings are essential as they can aid in evaluating credit default swaps and risk management strategies. A thorough understanding of primary commodity variation patterns can be invaluable in this context, assisting in more precise trend projections for the stock market, particularly in developing economies such as China. In our analysis of short-term dynamics, we noted that only stock market rates were significantly influenced by silver and oil prices. The ARDL analysis revealed that no other changes had long-term effects. 10.13039/100014337Furthermore, the analysis demonstrated that the equity index, supported by silver and oil prices and their fluctuations, stabilizes at a rate of 0.1 % of the dependent variable on a daily basis.

In our interpretation of the research, individuals involved in iron condor transactions can apply the results to mitigate risks in their investments. Participants in the market have the opportunity to utilize implied volatility contracts to oversee their stock portfolios, as these have been recognized as effective tools for managing risks. These contracts also act as a protective measure against unpredictable fluctuations in the oil, silver, and Chinese stock markets. Silver, known as a secure asset, not only offers security during financial and energy crises but also amid uncertainties related to health. Compliance with silver deposit regulations contributes to the stability of stock portfolios and economic prosperity, underscoring the importance of owners and authorities adhering to them. Investors need to make use of the information provided by volatility indices and promptly adjust to changes in oil production. In instances of heightened volatility in oil prices, investors should modify their stock exposure and decrease their holdings. To tackle the swift dissemination of information from oil markets to stock markets, it is necessary to enhance China's core stock market mechanisms, including the implementation of rapid response systems. Shareholders should consider cross-market discrepancies when formulating their strategies. 10.13039/100014337Furthermore, authorities should take proactive measures to support participants in the Chinese stock market and address any concerns related to potential shifts in the oil market.

### 5.1 Limitations of the study

• **Data Limitations**

The study's findings are based on data from China's security exchange from 1990 to 2022, which may limit the generalizability of the results to other regions or periods.

• **Scope of Analysis**

The study primarily focuses on the relationship between oil rates silver rates, and their impact on China's security exchange, potentially overlooking other relevant factors that could influence market volatility.

• **Model Complexity**

The empirical model used in the study may oversimplify the dynamics of the market by considering only a few variables, potentially neglecting the intricate interactions among various market indicators.

• **Market Specificity**

The study's focus on the Chinese market may restrict the applicability of the findings to global markets, as market behaviours and responses to commodity price fluctuations can vary significantly across regions.

• **Time Frame**

The study's analysis covers a specific time frame, and the long-term implications of silver and oil price volatilities may not be fully captured within this period.

### 5.2 Directions for future research

•Long-Term Effects of Silver and Oil Prices

Investigate the long-term effects of silver and oil price fluctuations on the stock market, considering how these changes impact investor behaviour and market stability.

• **Cross-Market Analysis**

Explore the interconnectedness between oil, silver, and security markets further to provide a comprehensive understanding for investors and policymakers.

• **Impact of Global Events**
Analyze how global events, such as pandemics like COVID-19, influence the volatility of commodity prices and stock markets, offering insights into crisis management strategies for future occurrences.
• **Policy Evaluation**

Evaluate the effectiveness of existing policies in managing market transitions and suggest improvements to enhance market resilience during periods of uncertainty.

• **Comparative Studies**

Conduct comparative studies across different regions or markets to assess the generalizability of the findings and identify region-specific factors influencing market volatility.

## Ethics approval and consent to participate

Not applicable.

## Consent for publication

All of the authors consented to publish this manuscript.

## Funding

This work was sponsored in part by the Key Project of 10.13039/501100012456National Social Science Foundation of China（No. 20AJL002）, Hunan Province Social Science Achievement Evaluation Committee Project（No. XSP20YBC275）and Hunan Provinc 10.13039/501100011788Philosophy and Social Science Planning Fund Project（No.22YBX018）.

## Data availability

We collected relevant data from World Bank open data available at https://data.worldbank.org/. For any further query on data, corresponding author at email address Bonnie_0313@126.com may be approached.

## CRediT authorship contribution statement

**Lei Zhou:** Writing – review & editing, Writing – original draft, Visualization. **Zhimin Gong:** Writing – review & editing, Writing – original draft, Visualization, Investigation, Conceptualization. **Lihui Tian:** Writing – review & editing, Visualization, Validation, Software, Data curation, Conceptualization. **Zaibi Chen:** Writing – review & editing, Writing – original draft.

## Declaration of competing interest

The authors declare that they have no known competing financial interests or personal relationships that could have appeared to influence the work reported in this paper.
